# The Efficacy of Orthodontics plus Implant Anchorage in Orthodontic Treatment: A Randomized Controlled Study

This article has been retracted.

**DOI:** 10.1155/2022/4049076

**Published:** 2022-05-30

**Authors:** Yuying Zhang, Keyue Li, Nan Li

**Affiliations:** ^1^Department of Stomatology of Jin Zhou Central Hospital, Jin Zhou 121000, China; ^2^Department of Medical Imaging of Jin Zhou Medical University, Jin Zhou1 21000, China; ^3^Neurology Department of Jin Zhou Central Hospital, Jin Zhou 121000, China

## Abstract

**Objective:**

To investigate the efficacy of orthodontics plus implant anchorage in orthodontic treatment.

**Methods:**

This randomized controlled study was conducted on 90 patients who had orthodontic treatment in our hospital between October 2019 and October 2020, and they were assigned to either a control group (*n* = 45) or an observation group (*n* = 45) via the random number table method. Patients in the control group received orthodontics while those in the observation group underwent orthodontics plus implant anchorage. The two groups were compared in terms of clinical indexes, efficacy, orthodontic state, adverse reaction rate, quality of life, and satisfaction.

**Results:**

After treatment, orthodontics plus implant anchorage led to lower gingival attachment level, gingival bleeding index, plaque index, and periodontal probing depth versus orthodontics alone (*P* < 0.05); orthodontics plus implant anchorage contributed to a higher efficacy versus orthodontics alone (91.11% vs. 73.33%, *P* < 0.05); orthodontics plus implant anchorage resulted in smaller molar displacement, larger protrusion distance of the upper central incisor, and larger inclination angle of the upper central incisor (*P* < 0.05); orthodontics plus implant anchorage was associated with fewer adverse reactions (4.44% vs. 26.67%, *P* < 0.05) and a higher quality of life scores versus orthodontics alone (*P* < 0.05); orthodontics plus implant anchorage yielded a higher satisfaction level versus orthodontics alone (95.56% vs. 66.67%, *P* < 0.05).

**Conclusion:**

The orthodontics plus implant anchorage offers a promising solution in orthodontic treatment. It is conducive to restoring dental indicators and improving quality of life and satisfaction. It is therefore worthy of application.

## 1. Introduction

Dental anomalies fall in the category of teeth, jaw, and craniofacial abnormalities caused by multiple factors in the oral cavity. Dental arch protrusions and tooth irregularities are common in dental anomalies, which adversely impact daily life and beauty [1]. Conventional orthodontic treatment is frequently used to resist the reaction force formed by the correction via absolute anchorage, but its efficacy remains poor due to its uncertainty and intense discomfort [2]. In recent years, implant anchorage has been extensively used in orthodontic treatment, with the advantages of low price, small size, and simple operation [3]. Orthodontic treatment is an orthodontic method that pushes the jaw or teeth to reach the ideal position. During the treatment, a certain reacting force will be generated that must be borne by the orthodontic anchorage. Therefore, the orthodontic anchorage is of great significance in orthodontic treatment. Oral cleaning after orthodontic treatment is extremely important. In this study, Jinzhijie gingival gargle was used to reduce the concentration of the inflammatory factor interleukin-6 in gingival crevicular fluid, improve various clinical indicators of orthodontic treatment, improve periodontal symptoms, inhibit the resorption of the alveolar bone, and promote the regeneration and recovery of periodontal tissues [4]. After basic periodontal treatment, Jinzhijie gingival gargle combined with orthodontic treatment can effectively control periodontitis, ensure straight teeth, eliminate jaw trauma, restore oral function, and maintain teeth outlook. Therefore, the present study aimed to explore the application of orthodontics plus implant anchorage in orthodontic treatment.

## 2. Materials and Methods

### 2.1. Baseline Information

This study was conducted on 90 patients who received orthodontics in our hospital between October 2019 and October 2020. Inclusion criteria were as follows: (1) patients aged 15 to 30 years; (2) patients who complied with all indications for orthodontics and implant anchorage surgery; (3) patients without gingivitis; (4) patients without oral mucosa disease; (5) patients without oral trauma and infection; (6) patients with no mental disorder but good compliance. Exclusion criteria were as follows: (1) patients with combined cancer; (2) patients with combined immune system disease; (3) patients with combined blood system disease; (4) patients with coagulation dysfunction; (5) patients who were pregnant or were breastfeeding. This study was reviewed and approved by the ethics committee of our hospital prior to commencing enrollment. All the patients voluntarily participated in the study and signed an informed consent form. According to the random number table, the patients were assigned to a control group (*n* = 45, orthodontics) and an observation group (*n* = 45, orthodontics combined with implant anchorage). After comparison, the two groups of patients showed similar baseline data as shown in Table 1. The research was approved by the Ethics Committee of Jinzhou Central Hospital, No. jz8819.

### 2.2. Research Methods

Patients in the control group received conventional orthodontic treatment. A facebow was used to strengthen the anchorage. After the patient wore the facebow, traction was performed on the teeth that needed orthodontic treatment. Every day, the patient wore a facebow for 8–12 hours of anchorage, and a transpalatal arch was inserted into the mouth to aid the correction.

Patients in the observation group underwent orthodontics combined with implant anchorage. First of all, local anesthesia was performed after patients completed mouthwashes, and the locations were marked where the implants were placed; the inside structure of the oral cavity was imaged and documented, including the form and structure of the root apex and the tissue structure around the implant; the mucosa of the alveolar site was cut to place the implant so as to prevent it from being involved in the mucosal tissue during the implantation; the implant was placed at 2-3 cm nearby the tooth root or the gingival site, with the implant perpendicular and slightly inclined to the bone surface during the implantation. After implantation, X-ray examination was performed to determine the relation between the implant and the tooth root, and antibiotics were given to keep the oral cavity clean and prevent oral infections. Subsequently, the implant with the traction hook was tightened using microtitanium nails. In addition, the rubber band was replaced regularly to the microtitanium nail that could be pulled out after counterclockwise rotation.

### 2.3. Support Treatment

During treatment, it is forbidden to use the mucoperiosteum to flap the gum of the affected tooth, so as to avoid the soft tissue at the corresponding mucous membrane being involved in the microimplant placement. After completing the operation, X-ray films were taken to ensure that the mini-implants and roots reached the ideal position. The implantation situation was observed, and antibiotics were given postoperatively to prevent infection. Implants were removed from the patient after orthodontic treatment. At the same time, Jinzhijie gingival gargle was given for dental care.

### 2.4. Observation Indexes

1. *Clinical Indexes*. After treatment, we examined the gingival attachment level and the periodontal pocket probing depth of the two groups, observed their tooth condition, and then evaluated plaque indexes and gingival bleeding indexes. The criteria for gingival bleeding indexes were as follows : 0 points indicated that the gum was healthy; 1 point indicated that there was a slight change in the gum color accompanied by mild edema, and it was considered mild if there was no bleeding during probing; 2 points indicated that the gum was red and brightly swollen, and it was considered moderate if there was bleeding during probing; 3 points indicated that obvious edema or ulcers existed at the gum, and it was considered severe if automatic bleeding appeared. Criteria for plaque indexes were as follows: 0 points indicated that there was no plaque in the gingival margin; 1 point indicated that there was thin plaque on the tooth surface of the gingival margin, which was invisible to the naked eye; however, the plaque was visible if the tooth surface was scraped with the tip of a probe; 2 points indicated that a moderate amount of plaque was seen on the gingival margin or adjacent surface; 3 points indicated that there was numerous soft dirt in the gingival sulcus or the gingival margin and adjacent surfaces.
2. *Clinical Efficacy.* (1) It was regarded as markedly effective provided that patients did not feel discomfort with regular teeth, normal molar occlusion, and normal anterior overbite, and coverage after treatment. In addition, their face shape had been greatly improved. (2) It was regarded as effective provided that patients did not feel discomfort with regular teeth and normal anterior overbite and coverage after treatment. In addition, their face shape had been improved. (3) It was regarded as ineffective provided that patients felt discomfort with relatively regular teeth and normal anterior overbite and coverage after treatment. In addition, their face shape showed no improvement [4]. Effective rate= (markedly effective + effective) cases/total cases × 100.
3. *Orthodontic Conditions*. We observed and recorded the orthodontic conditions of the two groups including molar displacement, the protrusion distance of the upper central incisor, and the inclination angle of the upper central incisor.
4. *Adverse Reactions.* After treatment, we observed and recorded the presence of edema, oral inflammation, root injury, and oral discomfort in the two groups. Adverse reactions rate = (edema + oral inflammation + root injury + oral discomfort) cases/total cases × 100.
5. *Quality of Life*. The self-made quality of life scale (with a full score of 100 points) in our hospital was used to assess the quality of life of patients who received orthodontic treatment before and after treatment. The higher the score, the better the quality of life.
6. *Patient Satisfaction*. The patients' satisfaction was assessed using questionnaires that composed of 10 items such as wearing comfort and aesthetics, with 10 points per item and a full score of 100 points. 90–100 points represented very satisfied level; 60–89 points represented satisfied level; <60 points represented dissatisfied level. Satisfaction rate = (very satisfied + satisfied) cases/total cases × 100%.

### 2.5. Statistical Analysis

All data analyses were performed using SPSS24.0 software. Measurement data are expressed as *x* ± *s* and compared using the *t*-test; count data are expressed as *n* (%) and compared using the *χ*^2^ test. Statistically significant difference was defined as *P* < 0.05.

## 3. Results

### 3.1. Clinical Indexes

After treatment, orthodontics plus implant anchorage led to lower gingival attachment level, gingival bleeding index, plaque index, and periodontal probing depth versus orthodontics alone (*P* < 0.05) (Table 2).

### 3.2. Clinical Efficacy

Orthodontics plus implant anchorage contributed to a higher efficacy versus orthodontics alone (91.11% vs. 73.33%, *P* < 0.05) (Table 3).

### 3.3. Orthodontic Conditions

Orthodontics plus implant anchorage resulted in smaller molar displacement, larger protrusion distance of the upper central incisor, and larger inclination angle of the upper central incisor (*P* < 0.05) (Table 4).

### 3.4. Adverse Reactions

Orthodontics plus implant anchorage was associated with fewer adverse reactions (4.44% vs. 26.67%, *P* < 0.05) (Table 5).

### 3.5. Quality of Life

Before treatment, no statistical significance was found in the comparison of quality of life scores between the two groups (*t* = 0.145, *P* > 0.05), whereas after treatment, there was a dramatic improvement in the quality of life of patients in both groups, with higher quality of life scores in the observation group (*t* = 5.742, *P* < 0.05) (Figure 1).

### 3.6. Satisfaction

There were 17 cases of very satisfied level, 13 cases of satisfied level, and 15 cases of dissatisfied level in the control group, while the numbers in the observation group were, respectively, 28 cases, 15 cases, and 2 cases; overall orthodontics plus implant anchorage yielded a higher satisfaction versus orthodontics alone (95.56% vs. 66.67%, *P* < 0.05) (Figure 2).

## 4. Discussion

In recent years, a growing number of individuals experience dental anomalies [5]. Though the leading causes of dental anomalies are complicated, the contributing factors such as trauma and disease have been identified [6]. Dental anomalies have detrimental impact on face shape, development of oral and facial muscle, pronunciation, oral health, chewing function, and mental state, resulting in a decline in the quality of life of patients [7].

At present, the mainstay for dental anomalies is orthodontics. Despite certain recovery effects, it is associated with many adverse reactions and high recurrence rate, thereby compromising the corrective outcome [8]. Therefore, it is urgent to optimize the treatment of dental anomalies in clinical practice. Nowadays, microimplant anchorage has been emerging in the orthodontic treatment and achieved remarkable clinical efficacy [9, 10].

In this study, after treatment, orthodontics plus implant anchorage led to lower gingival attachment level, gingival bleeding index, plaque index, and periodontal probing depth versus orthodontics alone; orthodontics plus implant anchorage contributed to a higher efficacy versus orthodontics alone (91.11% vs. 73.33%); orthodontics plus implant anchorage resulted in smaller molar displacement, larger protrusion distance of the upper central incisor, and larger inclination angle of the upper central incisor; orthodontics plus implant anchorage was associated with fewer adverse reactions (4.44% vs. 26.67%) and higher quality of life scores versus orthodontics alone; orthodontics plus implant anchorage yielded a higher satisfaction versus orthodontics alone (95.56% vs. 66.67%). These findings suggest that orthodontics plus implant anchorage might be a promising route for dental anomalies. In view of the large volume and poor stability of the common anchorage in conventional orthodontics, it will cause gingival bleeding, anchorage rotation, deformation, etc [11]. In addition, the nervousness, wearing discomfort, and poor coordination of patients hobble the safety of operation and treatment efficacy [12–14]. Encouragingly, the pronounced effectiveness of orthodontics plus implant anchorage can be attributed to the following: (1) Structurally, in orthodontics plus implant anchorage, the thread on the surface prevents synostosis and promotes the comfort in orthodontic treatment [15]. (2) The entire operation was simple and convenient, and anesthesia was not needed when the anchorage was removed in the later stage. The clot immediately filled in the space occupied by the anchorage after removal because of the small size of the implant anchorage, so as to prevent infection and accelerate the recovery of the wound [16]. (3) The stability reduced the damage to the oral cavity and the incidence of adverse reactions such as oral inflammation and tissue edema [17]. The implant anchorage was capable of loading in the early implantation due to its high safety and stability, and its strong endurance maintained traction, so as to ensure the treatment efficacy [18, 19]. (4) Since malocclusion and dental anomalies easily developed into periodontal lesion, the implant anchorage is conducive to reducing the periodontal disease through the improvement of correction, the tooth regularity, and the recovery of occlusion, thereby alleviating the periodontal pockets and facilitating the recovery of periodontal tissues [20, 21]. Eventually, the quality of life and mental state of patients would be greatly enhanced due to the improvement of appearance and quality of life. Jinzhijie gingival gargle is used to clear away heat, purify fire, detoxify, dispel wind, and remove dampness, with the main prescription of 12 herbal formulas including honeysuckle, skullcap, gardenia, *Sophora flavescens*, *Phellodendron*, solitary, mint, calamus, and mugwort. With cold herbs as the main method for clearing heat, purging fire, and detoxification and warm herbs as auxiliary to dispel wind, remove dampness, and dispel foulness, this medicine acts directly on the affected area, it can maintain and control the concentration and time of drug release and reduce the generation of bacterial resistance, with high effectiveness and safety profiles. Clinical observation found that Jinzhijie gingival gargle has a good auxiliary effect on orthodontic teeth, can effectively inhibit the occurrence of periodontitis, improve the local microecological environment of the periodontium, restore the periodontal ecological balance, and promote the restoration of periodontal tissue.

## 5. Conclusion

The orthodontics plus implant anchorage is a viable technique in orthodontic treatment, with higher effectiveness and safety profiles. It improves quality of life and satisfaction and is worthy of further popularization and application. However, this study failed to analyze the long-term effect of the combination of orthodontics and implant anchorage; therefore, it is elusive whether the long-term effect is stable, and the dental indicators remain in good condition for a long time. Hence, future studies with more long-term clinical data are required.

## Figures and Tables

**Figure 1:** Comparison of quality of life before and after treatment.

**Figure 2:** Comparison of satisfaction.

**Table 1:** Comparison of general materials.

Group	Gender (*n* (%))		Age ($\bar{x}$ ± *s*, years)	Orthodontic type (*n* (%))		
	Male	Female		Maxillary protrusion	Mandibular protrusion	Bimaxillary protrusion
Control group (*n* = 45)	27 (60.00)	18 (40.00)	24.19 ± 5.37	20 (44.44)	16 (35.56)	9 (20.00)
Observation group (*n* = 45)	25 (55.56)	20 (44.44)	23.84 ± 5.12	18 (40.00)	17 (37.78)	10 (22.22)
*t*/*χ*^2^	0.182		0.316	0.188		
*P*	0.670		0.752	0.910		

**Table 2:** Comparison of clinical indexes after treatment (*x* ± *s*).

Group	Gingival attachment level (mm)	Plaque index	Periodontal probing depth (mm)	Gingival bleeding index
Control group (*n* = 45)	3.35 ± 0.84	1.23 ± 0.37	2.89 ± 0.62	1.91 ± 0.57
Observation group (*n* = 45)	2.39 ± 0.68	0.69 ± 0.21	2.27 ± 0.43	0.54 ± 0.16
*t*	5.959	8.515	5.512	15.520
*P*	<0.001	<0.001	<0.001	<0.001

**Table 3:** Comparison of clinical efficacy (*n* (%)).

Group	Marked effectiveness	Effectiveness	Ineffectiveness	Effective rate
Control group (*n* = 45)	14 (31.11)	19 (42.22)	12 (26.67)	33 (73.33)
Observation group (*n* = 45)	25 (55.56)	16 (35.56)	4 (8.89)	41 (91.11)
*χ* ^2^				4.865
*P*				0.027

**Table 4:** Comparison of orthodontic conditions (*x* ± *s*).

Group	Molar displacement (mm)	Distance of the upper central incisor protrusion (mm)	Inclination angle of the upper central incisor (°)
Control group (*n* = 45)	6.37 ± 1.09	2.40 ± 0.75	14.08 ± 4.54
Observation group (*n* = 45)	3.24 ± 0.71	4.39 ± 1.28	26.15 ± 5.72
*t*	16.140	8.998	11.090
*P*	<0.001	<0.001	<0.001

**Table 5:** Comparison of adverse reactions (*n* (%)).

Group	Edema	Oral inflammation	Root injury	Oral discomfort	Incidence
Control group (*n* = 45)	3 (6.67)	2 (4.44)	3 (6.67)	4 (8.89)	12 (26.67)
Observation group (*n* = 45)	0 (0.00)	1 (2.22)	0 (0.00)	1 (2.22)	2 (4.44)
*χ* ^2^					6.154
*P*					0.013

## Data Availability

The datasets used during the present study are available from the corresponding author upon reasonable request.
